RETRACTED

# Impact of academic cheating and perceived online learning effectiveness on academic performance during the COVID-19 pandemic among Pakistani students

**DOI:** 10.3389/fpsyg.2023.1124095

**Published:** 2023-03-02

**Authors:** Aamir Abbas Malik, Mehdi Hassan, Muhammad Rizwan, Iqra Mushtaque, Tauqeer Ahmed Lak, Mussarat Hussain

**Affiliations:** ^1^College of Public Administration, Nanjing Agricultural University, Nanjing, Jiangsu, China; ^2^School of Education Sciences, Nanjing Normal University, Nanjing, Jiangsu, China; ^3^Department of Psychology, Bahauddin Zakariya University, Multan, Pakistan; ^4^Department of Sociology, University of Sargodha, Sargodha, Pakistan

**Keywords:** academic cheating, academic performance, Pakistan, COVID-19, students

## Abstract

**Objective:**

The study was conducted to examine academic cheating behaviors and perceived online effectiveness on academic performance during the period of COVID-19 among schools, colleges, and university students in Pakistan.

**Methodology:**

A cross-sectional research design was used in the current study. Convenience sampling was used to collect the data. The study included a total sample of *N* = 8,590 students, with males (*n* = 3,270, 38%) and females (*n* = 5,320, 61%) participating. The data was divided into three categories: high schools (*n* = 1,098, 12.7%), colleges (*n* = 4,742, 55.2%), and universities (*n* = 2,570, 32.1%). School students had an average age of (*M* = 15, SD = 4.65), college students had an average age of (*M* = 20, SD = 5.64), and university students had an average age of (*M* = 24, SD = 5.01).

**Result:**

The results indicated that 60% of students admitted to cheating during online exams most of the time; 30% of students admitted to cheating at least once during an online exam. The study found that students (from high school, college, and university) obtained higher grades in online exams as compared to physical exams. Furthermore, significant gender differences were found on the scales of online learning effectiveness in school, college, and university students (*t* = 2.3*, *p* = 0.05 vs. *t* = 4.32**, *p* = 0.000 vs. *t* = −3.3*, *p* = 0.04). Similarly, on the scale of academic performance, students have significant gender differences. Multivariate regression analysis confirms that students’ 26% academic performance was increased due to cheating (*F* (2, 8,588) = 16.24, *p* = 0.000). Students believe online learning is effective because academic grades are easily obtained.

**Conclusion:**

Cheating is more common and easier in online courses, according to more than half of respondents, and they take advantage of this. Academicians are heavily encouraged to develop morality and ethics in their students so that their institutions can produce ethical professionals for the educational community.

RETRACTED

## Introduction

Online education and evaluation have grown more common as a result of COVID-19. For the vast majority of online transfers, there is little time to ensure academic integrity (Zhao et al., 2022). Exams and papers are two of the most prevalent ways of evaluating students’ abilities (Comas-Forgas et al., 2021). The outcomes of these exams may have a significant impact on students’ future selves and professions, as well as their economic and social standing (Fontaine et al., 2020). Academic cheating may have surged during the COVID-19 outbreak, when institutions around the world moved to online instruction. This step has allowed students to finish their schoolwork using online resources, leading to more cheating. Students cheat more online because they believe it is easier than cheating in person (Lancaster and Cotarlan, 2021).

Academic cheating can be defined as deception, trickery, misrepresentation, or cheating (Fachruddin, 2017). Academic dishonesty and cheating are defined as student behavior that persuade the instructor that the student’s work is unique (Rehman and Waheed, 2014). Exam cheating (asking for help from classmates), plagiarism of other students’ work, collaboration on individual assignments, and the use of unlawful materials during examinations are all instances. Anderman and Won (2017) describe academic cheating as knowledge transmission, the use of aid, the exploiting of weaknesses, and the copying of answers or information. Cheating on homework, tests, and quizzes is common. Cheating, according to Sato and Ikeda (2015), includes giving, receiving, or receiving information during an exam or test, as well as obtaining material from unlicensed sources and skipping the evaluation method. Exam cheating is regarded as the most reprehensible act by both students and teachers (Chala, 2021). Student cheating, like academic cheating, has no universally accepted definition (McCabe et al., 2017). Numerous immoral behaviors intended to improve one’s or another’s “apparent” performance are frequently highlighted as evidence of student cheating.

Cheating is a major issue in education. The majority of research on cheating has been undertaken in Western countries, with an emphasis on its occurrence, causes, and definitions (Yazici et al., 2011; Byrne and Trushell, 2012). Few studies have looked into how individuals perceive cheating (Feinberg, 2009). Cheating’s incidence and frequency are determined by how seriously students take it. If a student believes that plagiarism on tests is unimportant, more occurrences will be recorded. Students who disagree with the morality of cheating are more likely to engage in it (Elias and Farag, 2010). Numerous surveys have been undertaken throughout the years to determine the prevalence of cheating in US universities and secondary schools. Two-thirds of college students and even more secondary school students admitted to cheating over the previous academic year (Lepp, 2017; Keskin and Uzuner, 2018; Mushtaque et al., 2021). The study found that 50 % of the 23,000 US high school students (grades 9–12) who participated had cheated on an exam the previous year (Jereb et al., 2017). Although investigations in other countries are uncommon, evidence indicates that cheating is not exclusive to a single nation or region (Ismail and Yussof, 2016). In one of the rare studies to compare exam cheating across nations, 7,200 university students from 21 countries revealed that rates and attitudes regarding exam cheating differed by nation, with less corrupt nations having the lowest levels of student cheating. Scandinavian nations were more trustworthy than most others (Teixeira and Rocha, 2010).

RETRACTED

Gender is a common indicator of deception. According to studies, men cheat more frequently and are more tolerant of infidelity than women (Hensley et al., 2013; Jereb et al., 2017). Despite the conclusion that gender has little direct influence on student cheating, other studies have found that social attributes associated with gender (such as shame, embarrassment, and self-control) account for differences in cheating behavior between males and females (Gibson et al., 2008; Modin et al., 2017). Another aspect connected with student cheating is academic achievement (most often operationalized as GPAs or grades). Students in lower grades are more likely to cheat than students in higher grades (Murdock and Anderman, 2006; Yang et al., 2013). Socioeconomic status (parents’ education, income, and occupation) has less of an impact on student cheating than previously thought (Kerkvliet, 1994). There has been little research into the relationship between migration and academic dishonesty. Çoban (2020) despite the fact that a study has not found a significant difference across ethnic groups, children who speak a foreign language may have more difficulty comprehending the curriculum (Mori, 2000). As expected, tolerant attitudes toward cheating increase its likelihood (Farnese et al., 2011). The view of cheating as unethical appears to have a greater impact on girls’ cheating behavior (Sarmiento and Manaloto, 2018). Students that have a low stress tolerance, a high risk tolerance, poor work ethics, and a lack of motivation are more likely to cheat (Sarmiento and Manaloto, 2018). Parental pressure and the desire to perform academically are also motivators for cheating students (McCabe, 2016).

RETRACTED

Cheating in school is acceptable when students believe their peers are cheating (McCabe, 2016). Cheating becomes normalized when a permissive culture emerges as a result of a shift in student attitudes; the more frequently students believe their classmates are cheating, the less blameworthy and morally wrong cheating is regarded to be (O’Rourke et al., 2010). Cheating is more common in schools that promote achievement and competitiveness than in schools that prioritize learning (Anderman and Koenka, 2017; Låftman et al., 2017). The ethos or culture of a school may influence a student’s proclivity to cheat.

Academic achievement has a substantial impact on teenagers’ and young adults’ professional growth (Wang et al., 2022). The current pendemic, according to studies, diminishes academic motivation and leads to learning loss among adolescents (Aboagye et al., 2020; Pitts and Kuhfeld, 2020). This is largely due to a lack of online learning preparation. According to PISA, the majority of 15-year-olds in 79 educational systems lacked the core skills needed to learn online (Khalilzadeh and Khodi, 2018).

## Aim of the study

Due to the COVID-19 outbreak, schools are now compelled to create alternatives to normal classrooms. Consequently, the majority of institutions, colleges, and schools in Pakistan have adopted online learning (Mushtaque et al., 2022). Whether or whether elementary and secondary school instructors are prepared, online education is expanding. After the proclamation of an emergency in Pakistan, online educations were implemented. Several colleges have transitioned from traditional on-campus education to hybrid (online and face-to-face) or online education. To continue education despite the COVID-19 pandemic, the majority of colleges have adopted online education. Concerns regarding academic dishonesty have been raised despite the benefits of online learning. According to research, the majority of students believe online learning makes cheating easier than traditional study methods (Hasri et al., 2022). In the current study we examined the students’ perception toward academic cheating during online classes and level of perceived effectiveness of online classes and their academic performance.

## Conceptual frame work

## Hypothesis of the research

*H1:* Academic cheating has the significant association with academic performance.

*H2:* Online learning effectiveness has the significant association with academic performance.

*H3:* Gender differences in academic cheating, online learning and academic performance.

RETRACTED

*H4:* Level of educational differences in academic cheating, online learning and academic performance.

## Methodology

This study analyzed students’ motivations for cheating, assessments of its severity, and impressions of online classes in order to analyze academic dishonesty in higher secondary schools, colleges, and universities. According to the study, cheating is increasingly common during school projects and assessments. This study looked into online exam cheating. A cross-sectional research design was used. Data was collected through convenient sampling.

### Participant selection and procedure

In the current study, we approached the schools, colleges, and universities to get the maximum number of students’ opinions. The data was collected from the two regions of Pakistan (Punjab and Sindh). Most of the authors belong to these regions of Pakistan. We approach public and private higher secondary schools, colleges, and universities. We obtain permission from the schools, colleges, and universities authorized and request that they circulate the online Google form to the student groups. After screening the data, incomplete forms were excluded and the statistical analysis was applied to the 8,590 participants.

### Ethical approval

The research approval was obtained from the Bahauddin Zikria University research committee and the research approval number is (ACD-22-231).

### Instruments

1. **Participant Information sheet:** In the current study, we took the data from secondary school students, college, and university students, so the participants’ gender, age, level of education, their grade during COVID-19, and grades in physical education classes were asked.
2. **Academic Dishonesty:** The academic dishonesty of students was assessed using a questionnaire based on literature and research. The study inquired about 10-items of exam cheating. The item scores range from 0 (never) to 2 (always; frequently). Cronbach’s alpha is 0.76, indicating strong inter-item consistency (Dejene, 2021). Students’ attitudes of cheating were also evaluated. Items were scored on a scale from 0 (cheat) to 5 (do not cheat; most serious). Lower perception indicates that pupils believe the behavior to be typical (acceptable). A Cronbach’s alpha of 0.72 indicates a high level of inter-item consistency. In addition, students were asked whether they had witnessed any instances of cheating (yes/no; Dejene, 2021).
3. **Perceived Online learning Effectiveness:** A 15-item scale was used in the current study to measure the students’ acceptance of online learning. This scale was developed by Lee et al. (2005). The scale has five domains (perceived usefulness, perceived ease, attitude, perceived enjoyment, and behavioral intensions). The reliability of the scale was 0.89.
4. **Academic performance:** Two-item questions were used in the current study to measure the students’ academic performance. Question 1: Grade, percentage, and CGPA prior to COVID-19 (face-to-face classes); and Question 2: Grade, percentage, and CGPA during COVID-19 (online classes).

RETRACTED

### Statistical analysis

In the current study, Descriptive statistics (frequency, mean and standard deviation) and inferential statistics; Pearson product moment correlation, independent sample *t*-test, multivariate analysis, and regression analysis were applied to the gathered data.

## Result of the research

In the current study, the total sample was *N* = 8,590, of which 61% were girls and 38% were boys. Further, the data was divided into three categories: high school students (1,098, 12.7%), college students (4,742, 55.2%), and university students (2,750, 32.1%). The mean age of the school students was (mean = 15), college students (mean = 20) and university students (mean = 24). During the online classes, school students (12.7%) revealed that they did not receive any lectures; their class teacher made a class group on Whatsapp and in that group they shared the assignments. Students at colleges and universities use Zoom (78.9%) and Team Meeting (8.2%) to take online classes (Table 1).

**Table 1:** Characteristics of the students (*N* = 8,590).

**Variable**	***F* (%)**	**M (SD)**
**Gender**		
Boys	3,270 (38.06)	
Girls	5,320 (61.93)	
**Age of the students**		
School		15 (4.69)
College		20 (5.34)
University		24 (5.01)
**Level of education**		
School	1,098 (12.7)	
College	4,742 (55.2)	
University	2,750 (32.1)	
**Online medium of instruction**		
Whatsapp	1,098 (12.7)	
Zoom	6,782 (78.9)	
Team meeting	710 (8.2)	

In Table 2, the prevalence of academic cheating is evaluated. 10% of students never engaged in academic cheating during online exams; 60% of students admitted to cheating during online exams most of the time; 30% of students admitted to cheating at least once during an exam.

**Table 2:** Prevalence of cheating during online learning.

Cheating statements	Never *F* (%)	Most of time *F* (%)	At least once *F* (%)
1. Copying classmates during an online exam	322 (3.7)	6,379 (74.2)	1,889 (21.1)
2. Permit others to use my online exam answers	340 (3.9)	5,795 (67.4)	2,455 (28.5)
3. Bringing study notes to an online exam	390 (4.5)	5,422 (63.1)	2,778 (32.3)
4. Sharing answers to an online exam with friends	512 (5.9)	5,304 (61.7)	2,774 (32.2)
5. Distributing electronic answer sheet to your friends	278 (3.2)	6,458 (75.1)	1,854 (21.5)
6. Write tips notes on bodily areas for cheating before the exam.	356 (4.1)	7,250 (84.4)	984 (11.4)
7. Falsifying reasons for missing an exam	671 (7.8)	5,386 (62.7)	2,533 (29.4)
8. Texting exam answers to friends through mobile devices	455 (5.2)	5,164 (60.1)	2,971 (34.5)
9. Text exam answers to friends through text message	590 (6.8)	5,189 (60.4)	2,811 (32.7)
10. Make excuses of internet connection	670 (7.7)	4,720 (54.9)	3,200 (37.2)

Table 3 depicts the differences between physical exam scores and online exam grades. On the online exam, no student from high school or college achieved <64%. Only about 0.5% of college students achieve a C grade. The ratio of grades on physical tests, on the other hand, is substantially different. The study found that online students engage in academic cheating.

RETRACTED

**Table 3:** Group comparison of academic grade (*N* = 8,590).

	Physical exam grades				Online exam grades				*f*	sig
	A (80%)	B (65%)	C <64	D <50	A (80%)	B (65%)	C <64	D <50		
(*n* = 1,098) School	324 (29.5)	479 (43.6)	175 (15.9)	120 (10.9)	988 (89.9)	110 (10.1)	–	–	5.6**	0.001
(*n* = 4,742) College	1,447 (30.5)	1,542 (32.5)	978 (20.6)	775 (16.3)	3,625 (76.4)	1,117 (23.5)	–	–	13.9*	0.26
(*n* = 2,750) University	1,049 (38.1)	1,203 (43.7)	343 (12.4)	155 (5.6)	1,435 (52.1)	1,300 (47.2)	15 (0.5)	–	3.2**	0.000

Significance **p < 0.001, *p < 0.05.

The gender differences at the school, college, and university levels are depicted in Table 4 above. The findings revealed that there were no significant differences in academic cheating between girls and boys during the COVID-19 online exam. Similarly, the university participants reveal that there is no statistical difference in academic cheating between boys and girls. While college students range significantly in the amount of academic cheating, boys are more likely than girls to engage in academic cheating on online exams. Online learning efficacy and academic achievement vary statistically between school, college, and university students.

**Table 4:** School, college and university wise gender differences on the study variables (*N* = 8,590).

School (*n* = 1,098)					College (*n* = 4,742)				University (*n* = 2,570)			
	Boys (*n* = 525) *M* (SD)	Girl (*n* = 573) *M* (SD)	*T*	Value of *p*	Boys (*n* = 2,988) *M* (SD)	Girl (*n* = 1,754) *M* (SD)	*t*	Value of *p*	Boys (*n* = 1,014) *M* (SD)	Girls (1,556) *M* (SD)	*t*	Value of *p*
AC	5.5 (4.5)	4.3 (4.0)	0.98	0.61	17.2 (11.5)	10.3 (9.1)	5.89**	0.000	9.2 (6.3)	9.0 (6.0)	1.28	0.93
OLE	17.3 (9.2)	14.6 (7.1)	2.3*	0.05	22.7 (8.2)	18.3 (6.7)	4.32**	0.000	15.1 (8.2)	19.6 (8.1)	−3.3*	0.04
AP	1.09 (0.8)	3.1 (1.9)	3.11**	0.000	5.4 (2.4)	7.1 (4.9)	4.29**	0.000	2.19 (1.5)	4.1 (2.3)	4.81**	0.000

AC, academic cheating; OLA, online learning effectiveness; AP, academic performance; *M*, mean; SD, standard deviation. **p < 0.01, *p < 0.05.

RETRACTED

On the basis of students’ academic cheating practices during online exams and online learning effectiveness, a multiple regression was performed to predict academic performance. The regression equation was found to be significant (*F* (2, 8,588) = 16.24, *p* 0.000), with an *R*^2^ of 0.014. The anticipated academic achievement of students is 0.25 plus 0.134 (online learning) plus 0.26 (academic cheating). Due to academic cheating, participants’ academic performance increased by 0.264. Both online exam cheating and online learning were significant indicators of academic performance (Table 5).

**Table 5:** Multiple linear regression analysis.

Model summary						
Model	*R*	*R* ^2^	Adjusted *R*^2^	SE of the estimate		
1	0.061^a^	0.014	0.014	0.88844		
**ANOVA** ^b^						
**Model**		**Sum of squares**	**df**	**Mean square**	***F***	**Sig.**
1	Regression	25.646	2	12.823	16.246	0.000^a^
	Residual	6845.779	8,588	0.789		
	Total	6871.425	8,590			
**Coefficients** ^b^						
**Model**		**Unstandardized coefficients**		**Standardized coefficients**	***T***	**Sig.**
		**B**	**SE**	**Beta**		
1	(Constant)	0.256	0.053		4.847	0.000
	Academic cheating	0.266	0.026	0.030	2.528	0.011
	Online learning	0.134	0.023	0.068	5.700	0.000

a Predictors: (constant), academic cheating, online learning.

b Dependent variable: academic performance.

## Discussion

The current study was meant to investigate the prevalence of academic cheating and the relationship between online learning effectiveness and students’ online academic achievement during the COVID-19 pandemic. According to the study’s findings, 60% of students acknowledged cheating most of the time, while 30% admitted to cheating at least once during an online exam. According to a prior survey, 80% of students participate in academic cheating. These findings are consistent with that finding. As evidenced by their lower estimations of the significance of academic cheating, the majority of students are more accepting of it (Dejene, 2021). Most students engaged in “sharing softcopies of answer sheets from friends,” “allowing others to cheat,” “opening books and notes to an online exam,” “texting solutions *via* mobile to friends,” and “providing answers to friends *via* signals” as the top five academic cheating techniques. The most prevalent kind of cheating that students admit to is copying and distributing their own exam papers. According to Pramadi et al. (2017), copying answers from peers is the most common method of cheating in high schools.

The study also looked at the opinions of male and female students to see if there were any differences in the severity of cheating between the sexes. Female students frequently rate the items as more serious than male students. In other words, women have demonstrated greater moral attitudes than men in relation to the vast majority of academic cheating practices. According to the study results, more than half of the respondents acknowledged cheating online because of its convenience and prevalence. They cheated by taking notes, utilizing a textbook, consulting with others, and copying answers from Google. Cheating was affected by a lack of expertise, higher grades, technical problems, the absence of monitoring, and exam stress (Dyer et al., 2020; Valizadeh, 2022). According to Holden et al. (2021), during COVID-19, seven million college students registered in at least one online course; if even a fraction of these students engaged in academic cheating, there would be tens of thousands of online cheaters per year. Many believe that online cheating is easier and more frequent than campus cheating. The results of the Holden study support the current study results; as we compared the campus-based exam grades and online exam grading, we found significant differences between the grades. During the campus-based exams, the ratio of grades varied, but in the online exams, students obtained A and B grades. Professors were asked about online vs. on-campus cheating. According to one-third of undergraduates, online classes encourage cheating. According to a survey, both professors and students agree that cheating on an online exam is easier (Erkut, 2020). Our second hypothesis was supported by the findings that online effectiveness measures were substantially associated with student cheating. In the current study, the student’s GPA was much higher on the online exam than on the in-person exam. GPA may influence a student’s desire for effective online learning. The result revealed a positive association between online effectiveness and academic performance.

RETRACTED

Although online learning has been encouraged in some areas, such as Pakistan, the school closures caused by the COVID-19 outbreak happened at an unsuitable time, delaying crucial academic activities and exams. Different assessment methods were adopted to maintain educational continuity. Assignments, portfolios, multiple choice questions, open book exams, and oral exams were employed as learning evaluations (Khan and Jawaid, 2020). Students in Pakistan were relieved to be enrolled in online classes because they were promoted based on the percentage of their prior grades and because they were permitted to utilize their books during tests (Mukhtar et al., 2020). According to Burgess and Sievertsen, internal assessments are given less weight in institutions due to the COVID-19 issue, resulting in cancelations. It should be highlighted that students who receive expected grades but receive actual ones have an effect on the job market (Burgess and Sievertsen, 2020). Universities that replace traditional tests with online assessments run the risk of committing moral and evaluative blunders. According to Alruwais et al., difficulties with online assessment include a lack of technical infrastructure, especially in developing countries; student unfamiliarity with hardware, software, and the assessment process; scoring issues; and difficulties with grading group work (Alruwais et al., 2018). Exam cheating by students needs additional precautions to ensure academic integrity. Examples include changing the format of electronic tests (using various forms, one-way examinations, fewer questions per page, and fewer time constraints), proctoring solutions, and changing the method of evaluation (oral exams, substituting exams with alternate modalities of assessment). Such initiatives will demand strategy, resources, and labor across the board. Grading and evaluation concerns may arise with remote E-exams, particularly in practical or clinical courses. Anti-plagiarism strategies and/or instruments must be updated (Basilaia and Kvavadze, 2020).

## Limitation of the study

There were some limitations to this investigation. First, memory bias could have influenced the data since students were asked to recall events they had performed or witnessed over the previous academic year that were online during COVID-19. Furthermore, because the responses were self-reported, they may be prone to social response bias due to the sensitive nature of the subject matter. However, the researcher’s promise of complete anonymity and emphasis on the necessity of authentic responses mitigated it. Despite its limitations, this study shed some information on how school, college, and university students perceive and engage in academic cheating during online learning.

## Conclusion

During the COVID-19 online exam in Pakistan, 60% of students admitted to cheating during online exams most of the time; 30% of students admitted to cheating at least once during an online exam. The study found that students obtained higher grades in online exams as compared to physical exams. Significant gender differences were found on the scales of academic cheating, online learning effectiveness and academic performance in school, college, and university students. Online learning has increased students’ opportunities to cheat and achieve easy grades, and grade comparisons show that students received higher grades on online exams. Due to the higher opportunity for academic cheating and the ease of gaining high grades, students perceived online learning effectiveness and showed high performance.

RETRACTED

## Data availability statement

The raw data supporting the conclusions of this article will be made available by the authors, without undue reservation.

## Ethics statement

The studies involving human participants were reviewed and approved by Bahauddin Zakariya University, Multan, Pakistan (SAR-20015). Written informed consent to participate in this study was provided by the participants’ legal guardian/next of kin.

## Author contributions

All authors listed have made a substantial, direct, and intellectual contribution to the work and approved it for publication.

## Conflict of interest

The authors declare that the research was conducted in the absence of any commercial or financial relationships that could be construed as a potential conflict of interest.

## Publisher’s note

All claims expressed in this article are solely those of the authors and do not necessarily represent those of their affiliated organizations, or those of the publisher, the editors and the reviewers. Any product that may be evaluated in this article, or claim that may be made by its manufacturer, is not guaranteed or endorsed by the publisher.
